The article "Mobile Technologies in the Early Detection of Cognitive Decline" was published in 2014. Journal: PLoS One.

# Mobile Technologies in the Early Detection of Cognitive Decline

**DOI:** 10.1371/journal.pone.0112197

**Published:** 2014-12-23

**Authors:** Michèle Allard, Mathilde Husky, Gwénaëlle Catheline, Amandine Pelletier, Bixente Dilharreguy, Hélène Amieva, Karine Pérès, Alexandra Foubert-Samier, Jean-François Dartigues, Joel Swendsen

**Affiliations:** 1 Univ. Bordeaux, INCIA, UMR 5287, Bordeaux, France; 2 CNRS, INCIA, UMR 5287, Bordeaux, France; 3 EPHE, Bordeaux, France; 4 CHU de Bordeaux, Bordeaux, France; 5 Univ. Bordeaux, ISPED, Centre INSERM U897, Bordeaux, France; 6 INSERM, ISPED, Centre INSERM U897, Bordeaux, France; University of Manchester, United Kingdom

## Abstract

The identification of biological and pathophysiological processes implicated in different forms of dementia is itself dependent on reliable descriptions of cognitive performance and capacities. However, traditional instruments are often unable to detect subtle declines in cognitive functions due to natural variation at the time of testing. Mobile technologies permit the repeated assessment of cognitive functions and may thereby provide more reliable descriptions of early cognitive difficulties that are inaccessible to clinic or hospital-based instruments. This assessment strategy is also able to characterize in real-time the dynamic associations between cognitive performance and specific daily life behaviors or activities. In a cohort of elderly rural residents, 60 individuals were administered neuropsychological and neuroimaging exams as well as a one-week period of electronic ambulatory monitoring of behavior, semantic memory performance, and daily life experiences. Whereas imaging markers were unrelated to traditional neuropsychological test scores, they were significantly associated with mobile assessments of semantic memory performance. Moreover, certain daily life activities such as reading or completing crossword puzzles were associated with increases in semantic memory performance over the subsequent hours of the same day. The revolution in mobile technologies provides unprecedented opportunities to overcome the barriers of time and context that characterize traditional hospital and clinical-based assessments. The combination of both novel and traditional methods should provide the best opportunity for identifying the earliest risk factors and biomarkers for Alzheimer's disease and other forms of dementia.

## Introduction

Despite considerable advances in molecular, functional and structural brain imaging techniques, their ability to identify biomarkers of the earliest phases of dementia has, to date, been unsuccessful [1]. This lack of progress is explained in part by the reliance of neuroimaging on reliable characterizations of cognitive performance as assessed through traditional clinical exams and neuropsychological assessment. In principle, detecting cognitive decline requires prospective testing over a period of years, but an individual's cognitive performance scores at any given assessment may fluctuate as a function of daily rhythms, emotion, stress and many other state-dependent influences [2], [3], [4], [5]. Due to this variance, subtle difficulties occurring in the earliest stages of dementia may be undetectable at the time of clinical examination, and their exploration through neuroimaging becomes feasible only for individuals having more salient cognitive deficits.

The article "Mobile Technologies in the Early Detection of Cognitive Decline" was published in 2014. Journal: PLoS One.

In addition to barriers to identifying anatomical correlates of early dementia, an additional challenge for research in this domain is the difficulty involved in isolating specific factors that may accelerate or slow cognitive decline. While diverse nutritional, behavioral and environmental factors have been linked to cognitive performance and to the risk of dementia [1], [6], a common assumption is that the benefits of specific daily life activities or lifestyles are seen cumulatively over periods spanning weeks to years. By contrast, recent research has shown that neural plasticity is far more dynamic than previously believed and that microstructural changes in the limbic system, especially the hippocampus, may be observable in the hours following certain activities [7]. The hippocampus plays an essential role in memory functions [8], [9] and is believed to be among the earliest brain structures affected in the course of Alzheimer's disease and other forms of dementia [10]. However, as neuropsychological assessments are most often conducted at one point in time or prospectively within a single environmental context, they cannot reliably link fluctuations in memory performance with specific daily life activities or experiences. This lack of information has consequences for brain imaging research, as the salience of potential biomarkers cannot be adjusted for the frequency of specific daily life variables that may constitute an important source of variance in imaging analyses. Knowledge of daily life behaviors associated with cognitive performance is also essential for the development of prevention strategies aimed at reducing the speed of cognitive decline and the risk of dementia.

Mobile technologies hold promise for overcoming these barriers by allowing for repeated assessments of cognitive functions and activities in real-time and across different contexts of daily life. These novel methods are increasingly applied in clinical research (NIH Medline Plus, 2011), and have been validated in a wide range of clinical populations, including within gerontology, psychiatry and neurology [11], [12], [13]. Cognitive performance scores derived through brief but repeated assessments may allow for more stable characterizations of cognitive difficulties very early in the course of dementia as well as provide more accurate information concerning the frequency and nature of daily life activities that influence cognitive performance. This investigation uses mobile cognitive assessments in healthy elderly individuals in order to: *i.* identify the neuroanatomical correlates of subtle deficits in cognitive performance; and *ii.* investigate the prospective association of specific activities with daily life cognitive functioning.

The article "Mobile Technologies in the Early Detection of Cognitive Decline" was published in 2014. Journal: PLoS One.

## Materials and Methods

### Participants

The current sample was drawn from a population-based cohort of 1002 elderly agricultural workers in rural France (the AMI cohort). Participants were randomly selected from the Farmer Social Security Registry and were at least 65 years of age. Study procedures were approved by the regional human research review board and all participants provided written informed consent. The inclusion criteria of the present study were having a 6^th^ grade reading level, no contraindication for MRI and no significant cognitive impairment or diagnosis of dementia (based on a neuropsychological evaluation by a psychologist, a clinical examination by a geriatrician and confirmation in a case consensus conference by three dementia specialists). Eighty-one individuals who met inclusion criteria were offered participation and 60 accepted.

### Procedures

At baseline inclusion in the cohort (September 2007 to March, 2009), participants were administered a neuropsychological test battery including the Mini-Mental Status Examination (MMSE; [14]) as an index of global cognitive performance, and the Isaacs Set Test [15] and Wechsler Similarities test (Wechsler D, 1981) to assess semantic memory capacities. A follow-up was conducted on average 2.5 years (SD = 0.21) later and included morphological MRI (Day 1). A subgroup of subjects completing MRI (n = 81) were also offered participation in a one-week period of ambulatory monitoring of cognition and behavior. Sixty individuals accepted these mobile assessments, which began on Day 1 immediately following the MRI exam and continued through Day 7, using a hand-held Personal Digital Assistant (PDA). In preparation for this ambulatory monitoring period, participants were trained in how to use the PDA, and then completed test assessments that were verified for accuracy and completeness with the research staff. The mobile assessments then occurred five times per day over a one-week period between 8:00 am and 10:00 pm, and with starting and ending times adapted to the participant's typical daily schedule. On average, each assessment required less than two minutes to complete, and responses were saved in a time-stamped database. The mobile assessment presented participants with questions of daily life experiences including activities and behaviors performed since the last assessment, their location, and their social company. Categories of activities were derived from previous EMA investigations [12], [13] and, for the purpose of analyses, were grouped into six broader categories that included chores (e.g. shopping, cleaning, cooking), socializing (telephone or in person), general sustenance or hygiene activities (e.g. eating, bathing, resting), physical activities (e.g. walking, gardening), passive leisure (watching TV) and intellectual activities (e.g. crossword puzzles, reading). In addition to questions administered at each electronic assessment, brief tests of semantic memory were randomly administered during two of the five daily assessments (resulting in 14 distinct tests over the assessment period). These mobile cognitive tests were modeled after the Wechsler Similarities test [13] and were pretested among cohort participants for feasibility and item comprehension. Each mobile test presented participants with a distinct list of 4 related objects or concepts, and then asked the individual to write into the PDA the broader category that described their association. Example test items included the presentation of the words “hammer, saw, screwdriver, and drill” (correct response: “tools”), or “Winter, Spring, Summer, and Fall” (correct response: “seasons”). The Isaacs Set Test was administered again in the same year as the MRI exam and mobile assessment.

The article "Mobile Technologies in the Early Detection of Cognitive Decline" was published in 2014. Journal: PLoS One.

#### MRI acquisition and data processing

Magnetic Resonance Imaging was performed using a 3 Tesla scanner (Achieva, Philips Medical System, The Netherlands) with a conventional quadrature head coil. Anatomical high resolution MRI volumes were acquired in transverse plan for each subject using a 3D MPRAGE T1 weighted sequence with the following parameters: 7-degree flip angle, TR = 8.2 ms, TE = 3.5 ms, matrix size 256×256, FOV 256 mm to cover the whole brain, yielding 180 slices and slice thickness of 1 mm, no gap, voxel size 1 mm3.

#### Cerebral volumetric assessments

An optimized procedure was performed to extract brain volumes using Voxel-Based Morphometry method [16], [17] using VBM5 toolbox (C. Gaser; http://dbm.neuro.uni-jena.de/vbm) of SPM5 framework. Total Intracranial Volume was computed as the sum of the GM, WM and CSF volumes.

#### Measurement of volumes of the hippocampus

FIRST is part of FMRIB's Software Library (FSL) (Oxford Centre for Functional Magnetic Resonance Imaging of the Brain Software Library, http://www.fmrib.ox.ac.uk/fsl) which performs subcortical brain segmentation using Bayesian shape and appearance models [18]. This method utilizes the shape and intensity variations of a structure for the purpose of automatically segmenting this structure. In our study, FIRST tool was applied to separately estimate left and right volumes of hippocampus. The segmentation was performed in two stages using affine transformations. In the first stage, the 3D T1 images are registered to the non-linear Montreal Neurological Institute (MNI) 152 standard space with 1×1×1 mm^3^ resolution using 12 degrees of freedom (DOF). The second stage uses an MNI subcortical mask of the hippocampus, followed by segmentation based on shape models and voxel intensities. The same registration procedure (12 DOF) is applied and a boundary correction method is used. Subsequently, volumes of hippocampus are calculated and all images of segmented hippocampus were visually checked for errors in registration and segmentation stages. In order to examine the specificity of the limbic system, the caudate nucleus was selected due to its capacity to be segmented by FIRST and its lack of implication in memory processes.

### Data analysis

In order to examine the association of standard neuropsychological test scores or MRI markers (hippocampal volume estimations with daily life activities and semantic memory performance), we used the Hierarchical Linear and Nonlinear Modeling (Raudenbush, et al., 2001) with Bernoulli models adjusted for age, sex, education, and Total Intracranial Volume (TIV, cm^3^). Intercepts-and-slopes-as-outcomes models, controlling for age, sex, and education were used to examine the prospective association of specific activities with subsequent cognitive performance.

## Results

The final sample (Table 1) was 45% female with a mean age of 75.06 years (SD = 4.66) and a mean baseline MMSE score of 26.97 (SD = 1.76, range = 22–30). Compliance of the sample with the repeated mobile assessments was high, with an average of 80.5% of the behavioral assessments and 78.6% of the semantic memory tests being completed over the assessment week. Scores for mobile semantic memory tests were significantly correlated with baseline neuropsychological test scores for Similarities (γ = 0.316, *t* = 2.096, p<0.05), as well as with the baseline Isaacs Set Test at 15 seconds (γ = 0.171, *t* = 4.921, p<0.001), 30 seconds (γ = 0.123, *t* = 5.370, p<0.001), and 60 seconds (γ = 0.069, *t* = 4.741, p<0.001).

The article "Mobile Technologies in the Early Detection of Cognitive Decline" was published in 2014. Journal: PLoS One.

**Table 1:** Demographic and clinical characteristics of the sample.

	%	Mean	SD
**Demographic variables**			
Age		75.06	4.66
% female	45.0		
Less than elementary school	26.7		
Elementary school	36.7		
More than Elementary school	36.7		
**Clinical variables**			
Baseline neuropsychological testing			
MMSE		26.97	1.76
Similarities		8.86	1.47
IST-15		28.39	5.13
IST-30		43.32	7.73
IST-60		64.05	13.17
Follow-up neuropsychological testing			
IST-15		28.02	6.56
IST-30		42.72	9.21
IST-60		62.68	15.36
Volumetric variables			
Total intracranial volume (cm^3^)		1484.12	176.89
Left HPC volume (mm^3^)		3456.37	457.09
Right HPC volume (mm^3^)		3620.58	459.20

MMSE (Mini-Mental Status Examination); IST (Isaacs Set Test).

### Cognitive performance and hippocampal volume

Adjusting for age, sex, education, and TIV, no significant associations were observed between left or right hippocampal volumes and neuropsychological tests scores obtained at baseline or at follow-up. However, the frequency of correct responses to the mobile semantic memory tests were significantly associated with volumes of both the left (γ = 0.0012, *t* = 2.950, p<0.01) and right (γ = 0.0013, *t* = 2.935, p<0.01) hippocampus (Table 2). This result was specific to this brain structure, as the same analysis using the caudate nucleus volume did not yield significant results. Fig. 1 illustrates these significant differences in mobile memory performance for individuals above or below the median hippocampal volume (3.453 cm^3^ for the left hippocampus; 3.613 cm^3^ for the right hippocampus).

**Figure 1:** Percentage of correct responses to mobile semantic memory tests as a function of hippocampal volume.

**Table 2:** Association of mobile semantic memory test scores with brain structure volumes.

	Left			Right		
Variable	Coefficient	SE	T-ratio	Coefficient	SE	T-ratio
Age	0.042	0.040	1.051	0.038	0.577	0.275
Sex	0.753	0.555	1.356	0.683	0.552	1.238
Education	1.017	0.282	3.606***	1.072	0.289	3.705***
Total intracranial volume	0.002	0.001	1.660	0.002	0.001	1.981
Hippocampus volume	0.001	0.000	2.950**	0.001	0.000	2.935**
Age	0.000	0.007	0.053	0.001	0.007	0.131
Sex	0.160	0.111	1.439	0.151	0.113	1.329
Education	0.183	0.064	2.871**	0.177	0.062	2.868**
Total intracranial volume	0.001	0.000	1.834	0.001	0.000	1.533
Caudate nucleus volume	−0.000	0.000	−0.848	−0.000	0.000	−0.382

**p<0.01,

***p<0.001.

### Cognitive performance and daily life activities

The mobile semantic memory scores were then examined relative to daily life activities and behaviors using time-lagged analyses. Socializing, general sustenance activities, physical activities and watching television had no effect on semantic memory performance over the subsequent three hours. However, intellectually stimulating activities (crossword puzzles, reading) were prospectively associated with increases in semantic memory performance over a subsequent three-hour period of the same day (γ = 0.893, *t* = 2.431, p<0.05).

The article "Mobile Technologies in the Early Detection of Cognitive Decline" was published in 2014. Journal: PLoS One.

## Discussion

Despite considerable progress made in dementia research, subtle declines in cognitive performance are often difficult to identify due to variation observed at the time of neuropsychological testing. This methodological limitation has slowed efforts to characterize biomarkers for the earliest stages of this disease, and the administration of tests within a single environmental context has also prevented investigation of the dynamic interplay of cognitive functions and daily life activities. The goal of the present study was to address these barriers by applying repeated mobile assessments of semantic memory performance and activity in the daily lives of elderly participants without dementia. The findings suggest that mobile technologies offer a new and powerful complement to traditional clinical tools for understanding the earliest stages of cognitive decline.

The feasibility of electronic ambulatory assessments has been previously demonstrated in healthy geriatric samples, as well as in elderly patients with neurological disorders [11], [12], [13]. However, while mobile technologies are increasingly used for *in vivo* cognitive testing, little is known about their contribution to the traditional methods used in psychiatry. Mobile cognitive assessments in the present study demonstrated strong concurrent validity with neuropsychological tests of semantic memory and verbal fluency, but were also able to characterize semantic memory performance over time and across contexts. For this reason, mobile performance scores may have a lower margin of error relative to single-assessment neuropsychological tests, and may therefore provide increased power to detect more subtle declines in cognitive capacities. Consistent with this possibility, hippocampal volume was significantly associated only with daily life semantic memory test scores, and not with traditional neuropsychological tests.

An important additional benefit of mobile technologies concerns their capacity to assess brief interactions among variables that may span periods of minutes to hours. In this way, memory performance scores were juxtaposed prospectively to discrete daily life behaviors. Semantic memory performance was found to significantly improve in the hours following intellectually-stimulating activities. This finding is consistent with the hypothesis that a regular practice of such activities may protect against cognitive decline [6] as well as with recent evidence demonstrating that brain microstructures may begin to change almost immediately following certain tasks or activities [7]. Despite the highly dynamic nature of neural plasticity, the literature to date documenting protective effects of specific activities or behaviors has focused on their cumulative association over substantially longer periods of time with the onset of salient cognitive problems or dementia [19]. Understanding the immediate impact of these daily life activities on the full spectrum of cognitive performance is inaccessible to traditional clinical methods but should provide empirical information that is currently lacking for prevention and early intervention strategies.

The article "Mobile Technologies in the Early Detection of Cognitive Decline" was published in 2014. Journal: PLoS One.

The focus of the present study on semantic memory is based on previous observations of the very early decline in this specific cognitive capacity among individuals who eventually developed Alzheimer's disease [20], [21], [22]. However, it is important to underscore that this illustration represents only one of many potential targets in the study of cognitive functions in daily life and of their corresponding biological and structural correlates using neuroimaging techniques. A more fundamental issue therefore concerns the methodological advances that can be obtained by pairing mobile technologies with other state-of-the-art tools administered in clinical and research contexts. The present findings should also be interpreted relative to the sample that was composed of retired agricultural workers with relatively low education levels. As it is likely that the sample's relatively low cognitive performance scores can be attributable in substantial part to lower education, the cohort should be considered as healthy elderly sample. While the sample size was sufficient for demonstrating a significant and specific association between mobile test scores and a previously-documented region of interest, it would likely be insufficient for full-brain exploratory analyses. Nonetheless, the apparent increased power of mobile assessments relative to traditional neuropsychological tests for a given brain structure, as well as its capacity to examine the dynamic interplay of cognition and behavior in real-time, demonstrates the promise of mobile technologies to the study of dementia risk and, more generally, as a complement to traditional clinical instruments.
